# Construction of Clinical Pathway Information Management System under the Guidance of Evidence-Based Medicine

This article has been retracted.

**DOI:** 10.1155/2021/4425449

**Published:** 2021-12-02

**Authors:** Xinyu Wang, Jie Chen, Fang Peng, Jingtai Lu

**Affiliations:** ^1^Department of Outpatient, PLA Rocket Force Characteristic Medical Center, Beijing 100088, China; ^2^Department of Medicine, Yangtze University, Jingzhou 434023, China; ^3^Department of Information Technology, PLA Rocket Force Characteristic Medical Center, Beijing 100088, China

## Abstract

This study focuses on clinical pathways guided by evidence-based medicine (EBM). With the clinical pathway as the center, the subjective and objective medical knowledge of medical staff are collected, and a clinical pathway management system guided by EBM is established through a unified process; user demand analysis; main considerations; implementation, evaluation, and monitoring of the clinical path; and dictionary maintenance, to help hospitals fully regulate medical behaviors. Next, the study displays the path access prompt box, area 1 management page, table management page, exit prompt box, mutation record page, doctor order interface, revocation of execution, and monitoring interface, and the system designed is compared with the Beijing Shankang Technology (ASK) clinical data management system in terms of user experience. The results showed that the reporting rate of medical adverse events in the system in this study was 0.21%, and the work efficiency was increased by 14%. In terms of users' satisfaction, the hospital managers' satisfaction was 84 ± 5.36%, and it was 95 ± 4.72% for medical staff and 88 ± 4.91% for system administrators, superior to the ASK system; the differences were statistically significant (*P* < 0.05). In conclusion, the clinical pathway information management system is in line with the working environment of medical staff, and the synchronous monitoring and management of medical quality are achieved through digital means, which can reduce the occurrence of medical adverse events and improve the work efficiency of medical staff.

## 1. Introduction

Before the 1980s, the medical research and practice were guided by traditional empirical medicine, which involved personal experience, textbooks, instructions from superior doctors, and some professional journals and literature [1]. With the passage of time, people gradually discovered the following problems in traditional medicine: the conclusions obtained from animal experiments are directly used in clinical practice, and their efficacy and safety cannot be determined; the popularization of observational studies or empirical results in the clinic leads to contradictions between clinical diagnosis and treatment methods; there are differences between actual treatment effects and clinical treatment effects that are inferred only based on the physiological/pathological mechanism of the disease [2, 3]. They all reflect the limitations under the guidance of traditional medicine.

In the early 1990s, Professor Guyatt first proposed the concept of evidence-based medicine (EBM). It was developed to scientifically diagnose diseases to formulate comprehensive treatment plans to improve clinical efficacy [4]. The development of health economics puts forward higher requirements for clinical medicine and how to make decisions with the massive medical evidence becomes a problem of great concern. All these factors promote the emergence and development of EBM [5]. EBM can better integrate the latest knowledge and technology in fields of epidemiology, information statistics, pharmacy, preventive medicine, and other disciplines and further extend the research to the fields of nursing, psychology, and economics [6]. The methodology of evidence production, conversion practice, and result evaluation developed later can handle various complicated events, providing relevant solutions for different industries. EBM can guide clinicians to use drugs in a mature and reasonable manner and make medical and health management more scientific. The clinical scientific research methods of EBM are mainly divided into design, measurement, evaluation, and rigorous evaluation, and its practical steps include problem-based learning, determining clinical problems, finding and collecting evidence, evaluating evidence, applying evidence, and proposing the best solution [7, 8]. Following the core idea of cautiousness and accuracy, EBM uses the latest research evidence available to formulate a treatment plan that best suits the patient's actual situation, plus the doctor's own professional skills and rich clinical experience, based on the patient's own pathological conditions and personal willingness. It represents the reform of medical education, the change of medical model, and the new definition of medical authority [9].

With the improvement of people's living standards, medical health attracts more and more attention; many potential diseases are discovered and diagnosed in time, and treatment plans for a certain single-factor disease are gradually mature and perfect. At the same time, the actual needs of patients and the requirements of medical care continue to expand. As a result, the work intensity of medical staff is increasing. Traditional medical care methods require a lot of time and manpower, and the clinical effects are not ideal. The rapid development of science and technology has contributed to the establishment of a mature, complete, and intelligent clinical information management system of high efficiency. On the one hand, it can manage the information of patients efficiently and monitor and control the physical condition of patients simultaneously; on the other hand, it can reduce human and material costs to a certain extent [10]. More importantly, clinicians and nurses can grasp the patient's condition changes, medication status, and treatment progress in real time, which can greatly reduce the difficulty and reduce the burden of clinical work. Besides, its clinical effects are more satisfying.

The meaning of clinical pathway is to construct a professional treatment mode or treatment plan by a group of members in medical and health institutions, including clinicians, medical experts, nurses, and hospital leaders, under the guidance of EBM so that patients are treated uniformly according to this mode from admission to discharge. Whenever a pathway is completed, the members of this group will analyze and evaluate it according to its results, check and compare the differences of each patient, and continuously improve and perfect the treatment plan [11]. The clinical pathway is a comprehensive treatment system using EBM as a guide to promote the management of disease diagnosis and treatment. It is aimed at standardizing medical methods, reducing the probability of differences, reducing costs in all aspects, and improving medical quality. Compared with treatment guidelines and treatment manuals, the clinical pathway is more concise in content, and the language is not obscure for reading and understanding. It can be used in a variety of disciplines and industry sectors. It is a standard diagnostic and treatment procedure for a specific disease or operation and values collaboration between each specialty in the treatment process [12].

However, there are also some problems in its treatment and management units. Some implementation units are one-sided and fail to involve all staff. First, when learning and formulating clinical pathways, the medical staff do not do in-depth thinking and do not agree on the goals and significance of the implementation of clinical pathways. Worse still, they do not know how to take the first step [13]. Second, the autonomy of medical care services is weakened, and the workflow of medical staff has become rigid. There are also some medical staff who repeatedly simplify the implementation of the clinical pathway, which will have a negative impact on the treatment of patients. In addition, there is also the idea that clinical pathways are only a formalized management method and have no practical value. Moreover, some people hold that the clinical pathway is just a reengineered diagnosis and treatment standard and it is meaningless [14]. Under these real problems, it is necessary to digitalize the information of clinical pathway and establish an information management system.

Clinical pathway information management system refers to an information system that uses network communication technology to collect, store, process, and transmit patient clinical information for use, with the ultimate goal of improving medical quality. The medical order processing system, laboratory system, and drug consulting system are all clinical pathway information management systems. Compared with hospital information system (HIS), the concept of clinical pathway information management system is completely different. HIS is developed to facilitate the work of the hospital's management personnel at all levels. Its purpose is to achieve information management of the information in all respects. The clinical pathway information management system mainly processes clinical information. It is oriented to clinical medical management and is patient-centric. The basic management unit is a clinical processing operation process based on medical knowledge, and the service subjects are medical staff. It aims to improve the quality of medical care and maximize the benefits of the hospital [15].

The innovation of this study lies in focusing on clinical pathway; under the guidance of EBM, a clinical pathway information system that can prompt in real time is established to standardize the medical behavior of the hospital, improve the quality of medical care, reduce the cost of the medical care process and of the patients, and improve the hospital's management level and efficiency.

## 2. Materials and Methods

### 2.1. Unified Process

The unified process is a process product developed by Rational. It is a framework that transforms user needs into a series of tasks to be completed by a software system. It specifies the steps to be taken to complete each task. The entire process uses Unified Modeling Language (UML) to complete the development planning of the software system [16], as shown in Figure 1. UML is a standard language for describing, visualizing, and documenting the products in the system used by users. It is developed on the basis of learning, extracting, and gathering all existing software modeling languages. Not limited by the software, UML can absorb a large number of modeling methods from other fields and has a solid and broad theoretical basis. It can be used not only for software modeling but also for modeling work in other fields [17]. It uses a series of graphic symbols to display the software model. These graphic elements have the advantages of simplicity, straightforwardness, and standardization and are friendly to the R&D personnel. The software model displayed by these graphic symbols can be straightforwardly understood and read. Because of its standardization, the accuracy and consistency of the model can be ensured.

### 2.2. Analysis of User Needs

User demand analysis refers to the investigation of actual user-oriented needs before system design and in the process of research, design, and development. It is the basis for system design, system improvement, and system maintenance. For an information management system, whether it can meet the actual needs of the users in all aspects is an important factor that determines its completeness [18]. The clinical pathway information management system, as management application software with the goal of standardizing the overall medical care process and improving the quality of medical care, needs to meet the actual needs of hospital managers as well as the clinical medical technicians. In addition, the needs of patients must also be taken into consideration. The clinical pathway can provide standardized medical documents to enhance communication between doctors and patients and reduce the conflicts between doctors and patients caused by information asymmetry. The clinical pathway information management system designed in this study is mainly oriented to four types of users, namely, hospital managers, medical technicians, patients, and system administrators.  Figure 2 shows the flow of the clinical pathway information management system.

### 2.3. Main Considerations

The clinical pathway information management system developed in this study is based on a full understanding of clinical pathways, and it uses existing medical resources for accurate monitoring and management of medical care. Then, the following factors should be considered.

The first is the guidance of knowledge related to clinical pathways. From a macro perspective, the essence of formulating clinical pathways is to collect opinions, discuss plans, and review and verify the results. It transforms the original tacit knowledge contained in the process into explicit knowledge, that is, the final clinical pathway knowledge. In the design of the clinical pathway information management system, EBM should be used as a guide to ensure that the final clinical pathway reserves more collective and personal experience and knowledge so that medical technicians can use this system more efficiently.

The second is to strictly regulate the formulation process of the clinical pathway, because the clinical pathway represents a standardized and strict medical care procedure, which requires a large number of surveys of doctors and patients and confirmation by industry experts and extensive collective discussions so that the clinical pathways developed are scientific and representative.

The third is the integration of clinical pathway information system and clinical information system. The clinical pathway is based on the clinical medical care work. Therefore, the design and development of the clinical pathway information system also need to be combined with the clinical information system so that the clinical events can be accurately monitored and managed. The integration of the clinical path information system and the clinical information system can also eliminate the need for medical staff to enter some repetitive information data, reduce time costs, and enhance the enthusiasm of medical staff.

The fourth is the analysis and statistics of the causes of the variation that may occur during the implementation of the clinical pathway. Compared with the clinical pathway, the traditional diagnosis and treatment model is rigid. The clinical pathway is in a dynamic process. It is superior to the traditional model in the learning ability. In the process of implementation by the medical staff, a large amount of information of each patient is collected, and modularized data processing analyzes actual clinical situations, which helps clinical pathway managers update the pathway content in a timely manner based on the feedback information.

### 2.4. Functional Division and Interrelationship Analysis of Clinical Pathway System

Out of consideration of the actual needs of the users, the clinical pathway information system is divided into the following main functions: setting and search of the knowledge base, conference management, formulation of clinical pathways, implementation of clinical pathways, and evaluation and monitoring of clinical pathways. In terms of the setting and search of the knowledge base, there are two requirements of the clinical pathway information system. One is that when the clinical pathway is formulated, the members of each responsible team need to record the most cutting-edge research conclusions on various professional medical websites and upload the web page link to the system for easy reference. The second is that the team members of each department can search for clinical pathway-related content in real time. This requires synchronous update of the knowledge base so that users can search related content through several keywords. At the same time, the clinical path information system needs to provide a channel for experts to modify settings so that users can intuitively understand the professional opinions of experts, as shown in Figure 3.

The requirements of the conference management are as follows. First, an organization must be established, including a leadership group and responsible groups for each department. Second, the learning of EBM and clinical pathway-related content is necessary, and a single training should last for at least 5 hours, with at least a total of 3 training times. In addition, the time and content of all conferences are recorded.

The formulation of clinical pathways is required to be serious, professional, and standardized. First, the inpatients and their families are investigated for general information. Second, the type of disease is determined. As per the International Classification of Diseases, the top 10 disease types are excluded one by one, and then common disease types are involved [19]. The system should be able to automatically provide the data of the International Classification of Diseases from the clinical information system. If not, it is necessary to set up a page (including the name of the disease and the code of the International Classification of Diseases) of the disease type. Third, the length of hospitalization and charging standards for the type of disease are identified. Responsible members of each department formulate the average length of hospitalization and charging standards for the disease, and if the patient has medical insurance, it will be determined according to the regulations of different medical insurances. The system needs to have the function of querying and counting the average length of stay and average expenditure of each single disease. Fourth, relevant information is sorted out. Responsible members of each department organize all personnel to participate in the meeting. The content of the meeting is to discuss and determine the collected disease types, the average length of stay and charging standards, the most cutting-edge scientific research conclusions of the disease, and the relevant content of the clinical pathway. Fifth, a meeting is held to determine the first draft of the pathway. Sixth, the system should be able to access the dictionary of doctor instructions and medical services so that the user can record the details of the daily clinical pathway. Seventh, the pathway table and implementation time are determined, and the system is required to have the classification confirmation and review functions of users with different permissions (Figure 4).

### 2.5. Implementation of the Clinical Pathway

The implementation of the clinical pathway needs to refer to the international disease classification code of the patient. If it exists in the disease list, the medical staff can work in accordance with the diagnosis and treatment standards set therein. The system needs to be combined with the doctor's workstation system. The user automatically obtains the clinical pathway form from the system and selects “whether to execute the pathway” according to the specific content (disease name, hospitalization days). If the user selects “Yes (execute),” the system will automatically execute according to the content in the table. If the user selects “No (do not execute),” the system will pop up the “Reason for non-implementation” prompt box for the user to fill in (Figure 5).

### 2.6. Evaluation and Monitoring of Clinical Pathways

The evaluation and monitoring of clinical pathways refer to the process of adjustment and improvement after medical experts make statistical evaluations of the clinical pathways. The clinical pathway is not rigid. It will be adjusted according to the actual situation. Under the authorization of the expert, the user will manage the newly added version of the clinical pathway table. Its main functions are summarized as follows. I. The system automatically stores the execution status of the clinical pathway and compares it with the expected goal. The content includes whether the plan is completed. If not, input reasons and measures are taken. II. It makes statistics on the execution of the terms in the pathway table, concerning path execution rate, mutation rate, and mutation category. III. If a case is discharged from the hospital, the system should have the function of automatically calculating the length and cost of hospitalization and, at the same time, compare the results with the set standards of a single disease. IV. It can be used to query the details of the mutation (Figure 6).

### 2.7. Dictionary and System Maintenance

Setting the content of the clinical path form requires a strict and standardized doctor order system to support it, and the condition of the disease also needs to have its corresponding clinical information system doctor order dictionary as a reference. In addition, it requires the maintenance of a dictionary for the names of single diseases, the maintenance of international disease classification codes, the types of medical instructions, and the reasons for path variation (Figure 7).

### 2.8. Database Design

The database is the basis of the information system. It integrates the massive data into the information system according to a specific model and has storage, maintenance, and query functions, so that the information system can quickly, timely, and accurately retrieve the information needed from the database. The content of database design mainly includes four aspects: database requirement analysis, database conceptual structure design, database logical structure design, and database structure realization.

The content of the data demand analysis includes the clinical pathway table, the clinical pathway and clinical information system interface table, and the monitoring disease standard name table. The conceptual structure design is based on demand analysis and lays the foundation for the future logical structure design. This research uses UML for the database conceptual structure design. The logical structure of the database is an information structure independent of the actual data model, which must be transformed into a logical structure before the design. After the logical structure of the database is designed, the system connects to the Oracle Database, performs data modeling through the “Enterprise Manager,” and automatically selects and configures the database according to the different selections.

### 2.9. Comparison of Two Systems

After the system is set up and tested, to evaluate the user experience, another clinical information system is selected for comparison. After communication, First Affiliated Hospital of Yangtze University used the clinical data management system developed by Beijing Shankang Technology (ASK), and PLA Rocket Force Characteristic Medical Center used the clinical pathway information management system developed in this study. The use time was 6 months, and the subjects included hospital managers, medical technicians, administrative personnel, and logistics personnel.

### 2.10. Statistical Analysis

All data were statistically analyzed using SPSS 24.0 software. Measurement data are expressed as mean standard ± deviation ($\bar{x}$ ± *s*). Count data is expressed as a percentage. The comparison between multiple groups uses one-way analysis of variance. *P* < 0.05 indicates that the difference is statistically significant.

## 3. Results

### 3.1. Path Admission Prompt

After entering the system, the clinician clicks Western Medicine Diagnosis Entry-Enter Diagnosis in turn. If there is a clinical pathway that matches the diagnosis, an admission prompt box will pop up, as shown in Figure 8.

### 3.2. Entry into the Clinical Pathway

After logging in, the clinician can enter the “Clinical Path Management” menu after selecting a patient.  Figure 9 is the access area 1 management page, which displays the current patient's basic information and medical treatment information. Besides, the current pathway information and the stage information of the patient are also displayed. The “Table Display” page will display the clinical pathway content, as shown in Figure 10.

### 3.3. Exiting from the Clinical Pathway

On the entry and exit page, the clinician clicks the “Exit” button to exit the current page, as shown in Figure 11.

### 3.4. Variation Record

On the entry and exit page, the clinician clicks the “Mutation record” button to enter the disease mutation record page, as shown in Figure 12.

#### 3.4.1. Medical Order Issuance

On the “Doctor's Order Entry” page, the clinician clicks the “Clinical Path” button to access the clinical pathway table of the patient, as shown in Figure 13.

### 3.5. Revocation of Execution

After entering the “Clinical Path Cancellation Execution” menu, the clinician selects the items that have been executed in the “Main Diagnosis and Treatment Work” column, and then the “Cancel Diagnosis and Treatment Records” interface pops up. Next, the clinician selects the terms that need to be canceled and clicks the “OK” button to complete the cancelation action, as shown in Figure 14.

### 3.6. Monitoring Interface

After the system administrator logs in, the monitoring interface is shown in Figure 15.

### 3.7. Comparison Results of the Two Systems

After the system was set up and tested, to evaluate the user experience, another clinical information system was selected for comparison. The results are shown in Figure 16. The reporting rate of adverse medical events under the ASK system was 0.43%, and the reporting rate of the system in this study was 0.21% (*P* < 0.05), which indicated that the incidence of adverse medical events under this research system was low. The user efficiency of the ASK system was increased by 9%, while the user efficiency was improved by 14% for the system in this study (*P* < 0.05). In terms of user satisfaction, hospital managers' satisfaction with the ASK system was 78 ± 5.32%, that of the medical staff was 74 ± 4.83%, and that of system administrators was 76 ± 4.96%. The user satisfaction with this system was 84 ± 5.36%, 95 ± 4.72%, and 88 ± 4.91%, respectively. The differences between the two systems were statistically significant (*P* < 0.05).

## 4. Discussion

EBM refers to the combination of the doctor's personal clinical experience and professional knowledge and skills with the best evidence of existing clinical research to make clinical diagnosis, in response to specific problems that need to be solved in the clinic [20]. EBM and traditional medicine are different in research methods and involved technologies. Traditional medicine is mainly based on empirical medicine. The so-called empirical medicine is based on the doctor's own understanding of the basic knowledge of the disease and the accumulation of personal clinical experience, combined with the analysis of clinical data [21]. EBM is not and cannot replace empirical medicine. It mainly emphasizes that any medical decision-making process should be based on the scientific research and scientifically collected evidence [22].

Clinical pathway is a procedural and standardized diagnosis and treatment plan based on EBM, aimed at standardizing medical service behaviors and reducing recovery delays and resource waste, so that patients can obtain the best medical care services [23, 24]. The clinical pathway emphasizes completeness and cooperation. It means that all members who provide medical care services jointly formulate the treatment content and execution time. In clinical practice, the patient is the center, and the work of multiple departments, including professional departments and administrative departments, is integrated; it emphasizes horizontal contact and communication between departments. The clinical pathway is not a standard of behavior, but a kind of guidance or advice, and does not deprive the doctor of autonomy [25]. It proposes the best diagnosis and treatment plan discussed and approved by experts, which reduces the difference in treatment effects due to different levels of doctors and protects the interests of patients. When using clinical pathways, doctors are also allowed to make corresponding adjustments according to the actual situation of the patient.

EBM has a close relationship with clinical pathways. At the beginning of the 21st century, there was literature that specifically mentioned the relationship between the two. It is believed that the two have the same goal of serving medical care, and they coordinate with each other to promote the development [26]. In recent years, with the advancement of clinical pathways, the integration of clinical pathways and EBM has expanded to the combination of hospital knowledge management and clinical pathways. The role of clinical pathways is obvious, but the difficulty of implementing the clinical pathways is also very obvious. The record process is cumbersome, the clinical pathways are still difficult to promote in primary hospitals, and the types of diseases recorded are also very limited. How to easily and quickly record all the content required by the clinical pathway and continuously improve work efficiency is an urgent and important task for the majority of medical workers.

In this study, with the clinical pathway as the center, the subjective and objective medical knowledge of medical staff are collected, and a clinical pathway management system guided by EBM is established through a unified process; user demand analysis; main considerations; implementation, evaluation, and monitoring of the clinical path; and dictionary maintenance, to help hospitals fully regulate medical behaviors. The third section of this study displays the path access prompt box, area 1 management page, table management page, exit prompt box, mutation record page, doctor order interface, revocation of execution, and monitoring interface, and the system designed is compared with the ASK clinical data management system in terms of user experience. The results showed that the reporting rate of adverse medical events under the ASK system was 0.43%, and the reporting rate of the system in this study was 0.21% (*P* < 0.055), which was similar to the research results of Luo et al. [27]. The user efficiency of the ASK system was increased by 9%, while the user efficiency was improved by 14% for the system in this study (*P* < 0.05). In terms of user satisfaction, hospital managers' satisfaction with the ASK system was 78 ± 5.32%, that of the medical staff was 74 ± 4.83%, and that of system administrators was 76 ± 4.96%. The user satisfaction with this system was 84 ± 5.36%, 95 ± 4.72%, and 88 ± 4.91%, respectively. The differences between the two systems were statistically significant (*P* < 0.05), which was consistent with the research conclusions of Tippenhauer et al. [28]; that is, the clinical pathway information management system can standardize the hospital's medical behavior, optimize the quality of medical care, reduce the cost of medical services and hospitalization, and improve the level of hospital management.

## 5. Conclusions

In the study, a clinical pathway information system is designed under the guidance of EBM to improve the clinical diagnosis abilities of medical staff. The system is integrated with the clinical information management system to obtain faster and more accurate data support and to effectively use digital means to fully intervene in the medical process. It is found to have a significant effect on reducing the occurrence of medical adverse events and improving work efficiency. The limitation of this study is that the combination of EBM and hospital clinical pathway has not been tested in depth, and further theoretical discussion is needed in a later stage.

## Figures and Tables

**Figure 1:** Schematic diagram of the unified process.

**Figure 2:** Flow chart of clinical pathway information management system.

**Figure 3:** Functional division and interrelationship analysis of the clinical pathway system.

**Figure 4:** The development process of clinical pathways.

**Figure 5:** The implementation flow of the clinical pathway.

**Figure 6:** Evaluation and monitoring of clinical pathways.

**Figure 7:** Maintenance of the clinical pathway.

**Figure 8:** Path admission prompt diagram.

**Figure 9:** Management page of access area 1.

**Figure 10:** Pathway table page.

**Figure 11:** Exiting from the clinical pathway.

**Figure 12:** Variation record page.

**Figure 13:** The doctor's order interface under the current clinical pathway.

**Figure 14:** Cancelation execution interface.

**Figure 15:** Monitoring interface.

**Figure 16:** Comparison of the two systems. (a) Adverse event reporting rate and work efficiency improvement rate; (b) user satisfaction. *∗* means that the difference was statistically significant compared with the ASK system (*P* < 0.05).

## Data Availability

The data files are available from the corresponding author upon reasonable request.
